The article "Protective Effect of Effective Components of Coreopsis tinctoria Nutt on Retinopathy of db/db Diabetic Mice" was published in 2021. Journal: Evid Based Complement Alternat Med.

# Protective Effect of Effective Components of *Coreopsis tinctoria* Nutt on Retinopathy of db/db Diabetic Mice

**DOI:** 10.1155/2021/9948609

**Published:** 2021-10-14

**Authors:** Li Hui, Yang Tao, Mao Xinmin

**Affiliations:** ^1^Central Laboratory of Xinjiang Medical University, Urumqi 830011, China; ^2^College of Traditional Medicine, Xinjiang Medical University, Urumqi 830011, China

## Abstract

**Objective:**

Diabetic retinopathy (DR) is one of the main diabetic microvascular complications in clinical practice, which features a complicated mechanism and insignificant efficacy. Therefore, it is urgent to find effective drugs. Xinjiang *Coreopsis tinctoria* Nutt is a rare alpine wild plant with unique effects and extremely high medicinal value. Preliminary studies have shown that it can reduce elevated blood sugar, unhealthy lipids, and antioxidants. This study was intended to investigate the protective effect of the effective components of *Coreopsis tinctoria* Nutt on the retinopathy of db/db diabetic mice and provide experimental basis for exploring the efficacy of *Coreopsis tinctoria* Nutt and the development of new drugs for the treatment of DR.

**Method:**

The db/db diabetic mouse models were used, and the effective components of *Coreopsis tinctoria* Nutt were obtained from *Coreopsis tinctoria* Nutt using macroporous resin enrichment method after alcohol extraction. These mice were divided into the normal group, model group, and high-dose Coreopsis *tinctoria* Nutt groups, the positive drug metformin group, and the metformin and *Coreopsis tinctoria* Nutt combination group. After these db/db type 2 diabetes mouse models were intervened for 10 weeks, their weight, blood sugar, glycosylated hemoglobin, serum MDA, SOD, and other indicators of each group were tested, and the expression changes of VEGF, ICAM1, PEDF, Bcl-2 in mouse retina were observed by immunohistochemistry method.

**Result:**

The effective components of *Coreopsis tinctoria* Nutt were obtained using macroporous resin enrichment method after alcohol extraction, which were mainly comprised of chlorogenic acid, flavone mariside, mariside, dicaffeoyl quinic acid, and flavone oxanine, with a total content of 532.82 mg/g, and the total flavonoid content of 330 mg/g. The effective components of *Coreopsis tinctoria* Nutt significantly reduced blood sugar and glycosylated hemoglobin and improved oxidative stress levels in db/db diabetic mice. Meanwhile, they reduced the expression of VEGF and ICAM1 in retinopathy and increased the expression of Bcl-2 and PEDF. The combination of *Coreopsis tinctoria* Nutt and metformin has the most significant effect.

**Conclusion:**

*Coreopsis tinctoria* Nutt can prevent and treat early diabetic retinopathy by affecting the expression of retinopathy-related factors.

## 1. Introduction

Diabetic retinopathy (DR) is one of the common and serious microvascular complications of diabetes, which is the manifestation of metabolic disorders and abnormal changes in the blood system in the retina caused by the body's endocrine system. The main clinical symptoms are retinal hemorrhage, exudation, abnormal internal circulation, macular edema, neovascularization, vitreous hemorrhage, and traction retinal detachment, which ultimately lead to severe visual impairment. DR is the leading cause of visual impairment in the adult population of developed countries [1], and its incidence in China has recently also increased year by year [2]. Therefore, the research on the pathogenesis of DR and the exploration of effective preventive drugs has been highlighted issues [3]. Xinjiang *Coreopsis tinctoria* Nutt is an annual herb of the genus *Coreopsis* in Compositae with unique efficacy and medicinal value as a rare wild alpine plant. In the folk, *Coreopsis tinctoria* Nutt is often quoted as flower tea by the local minorities. It has the functions of clearing away heat and detoxification, invigorating stomach and spleen, promoting blood circulation and removing blood stasis, reducing dampness and stopping dysmenorrhea. It mainly contains flavonoids, volatile oils, amino acids, saponins, polysaccharides, chlorogenic acid, and other components [4]. The study results of Mao [5] showed that the extract of *Coreopsis tinctoria* Nutt can reduce blood glucose and improve blood lipid in experimental diabetic mice, and its mechanism may be related to the recovery of islet *β*-cell function and the promotion of insulin secretion. The study results of Lan [6] showed that the alcohol extract of *Coreopsis tinctoria* Nutt could significantly improve the dyslipidemia of diabetic rats. db/db mice was a mutant line screened from C57BL/6J mice by Jackson Laboratory in 1966. Due to the recessive leptin receptor gene defect on the autosome, short-chain leptin receptor Ob/Ra replaced long-chain leptin receptor Ob/Rb, leading to spontaneous diabetes. The homozygous (db/db) mice born after four weeks gradually show the characteristics such as obesity, elevated blood sugar blood fat, and insulin resistance. After 8–12 weeks, blood sugar will continue to rise, until chronic complications and islet B cell function failure or death around 10 months occur. This disease process is very similar to the process of human development of type 2 diabetes. Therefore, it is currently an ideal animal model for the study of human type 2 diabetes mellitus [7, 8]. The previous study indicates that the ethyl acetate extract of *Coreopsis tinctoria* Nutt may play a certain protective effect on diabetic retinopathy by downregulating the expressions of VEGF and ICAM1 [9]. In this study, the effective components of *Coreopsis tinctoria* Nutt were obtained by the method of alcohol extraction with macroporous resin enrichment to intervene in the db/db diabetic mouse model, and the improvement of the blood glucose and overall oxidative stress state of the mice after the intervention was observed. With retinopathy as the entry point, the effect of *Coreopsis tinctoria* Nutt on the expression of related factors of diabetic retinopathy in mice was observed to preliminarily discuss the protective effect of Xinjiang *Coreopsis tinctoria* Nutt on diabetic retinopathy.

## 2. Materials and Methods

### 2.1. Experimental Animals

Six-week-old spontaneous diabetic db/db mice were selected for the diabetes model group, weighing 30 ± 2 g, and the normal male mice of the same age with db-BLKS background were selected for the control group, weighing 16 ± 2 g. All the mice were raised in the SPF barrier environment of the Animal Experiment Center of Xinjiang Medical University, which simulated natural day and night conditions, with daytime relative temperature of (21 ± 2)°C, relative humidity of 40%∼45%, daily sunshine time of 12 hours, and free feeding and water intake. After two weeks of adaptive feeding of db/db mice, their tail tip blood was taken to measure the fasting blood glucose (FBG), and the model >7.0 mmol/L. The study was authorized by the Institutional Animal Care and Use Committee of First Affiliated Hospital of Xinjiang Medical University (Approval No.: IACUC-20140304011).

In order to minimize the experimental error caused by individual animal differences, the mice of the model and normal control groups were purchased from the same company, and the model mice were in the same batch.

### 2.2. Medicinal Material Extraction

#### 2.2.1. Alcohol Extraction Method

The *Coreopsis tinctoria* Nutt is produced in Minfeng County, Hotan Prefecture, Xinjiang. A multifunctional extractor was used for the process amplification extraction of the *Coreopsis tinctoria* Nutt. An appropriate amount of the *Coreopsis tinctoria* Nutt raw material was weighed into the extraction tank of the multifunctional extraction unit, added with the corresponding volume of 55% ethanol at a material-to-liquid ratio of 1 : 15, which was soaked for 12 hours, and then heated and extracted using a continuous reflux device for 2.5 hours, with the heating temperature set at 45°C. After the extract was concentrated by a rotary evaporator, it was put into a vacuum drier at a temperature of 55°C and a vacuum degree of 0.07 MPa, grounded into fine powders, and sealed in bags at −20°C for use after they completely dried.

To ensure the reproducibility of experimental results, the reagents and positive drugs used in the experimental process were all from the same batch and company. The *Coreopsis tinctoria* Nutt medicinal materials were all from the same harvest time and the same place of production. The effective components were prepared by a unified extraction method, which could only be used after passing the testing of consistency between the quality standards and content.

#### 2.2.2. Purification with Macroporous Resin

At the sampling concentration of macroporous resin of 20 mg/mL, the sample was added into the macroporous resin column for 12-hour adsorption and then eluted with four column volumes of distilled water at a flow rate of 3 BV/h, followed by four column volumes food grade ethanol with a concentration of 75% for elution at an elution rate of 3 BV/h, and the eluent was collected finally. The collected eluent was concentrated via a vacuum rotary evaporation equipment till thickness and then poured into a ceramic evaporating dish, which was put in a vacuum drier for drying with an appropriate amount of silica-gel drier. After the ethanol was evaporated dry, the powders were scraped out and stored at −20°C for later use.

#### 2.2.3. TLC Detection Method

The powders obtained from *Coreopsis tinctoria* Nutt after alcohol extraction with macroporous resin enrichment were mixed with distilled water into a solution with a concentration of 15 mg/mL, which was used to sample the spot plate via an automatic sampler, with the sample volume of 10 ul, conducted in the ternary system of toluene: ethyl acetate: formic acid = 9 : 7 : 3.

#### 2.2.4. HPLC Method

Chromatographic column: shim-pack vp-ODS (150 mm *∗* 4.6 mm, 5 um); elution flow rate 1.0 mL/min; detection wavelength: 280 nm; column temperature: 35°C; sampling volume: 10 uL; mobile phase: phase A 0.5% formic acid solution, phase B acetonitrile. Elution method: gradient elution: elution with 95%–80% mobile phase A and 5%–20% mobile phase B for 60 minutes, then elution with 80%–60% mobile phase A and 20%–40% mobile phase B for 50 minutes, and finally elution with 60%–95% mobile phase A and 40%–5% mobile phase B for 20 minutes.

### 2.3. Model Confirmation and Group Intervention Methods

After two weeks of adaptive feeding of db/db mice, their tail tip blood was taken to measure the FBG; the model >7.0 FBG was established; the mice were administered intragastrically. Except for the normal group (NG), the diabetic mice were divided into five groups: the model group (diabetic control group, DC) as a control without administration, the positive drug control group (DC + metformin group, DC + M) given the positive drug metformin, with the doses of 180 mg/kg, high and low dose effective components of *Coreopsis tinctoria* Nutt (DC + effective components of *Coreopsis tinctoria* Nutt group, DC + EC), with the doses of 300 mg/kg (DC + EC300) and 150 mg/kg (DC + EC150) respectively, and the metformin plus *Coreopsis tinctoria* Nutt combination group (DC + M + EC) with the doses of 180 mg/kg of M and 150 mg/kg of EC to observe the combination efficacy of traditional western with Chinese medicines. The drug was dissolved in 0.1 M citric acid and 0.1 M sodium phosphate solution and then administered by gavage. The mice were weighed weekly, and blood was collected from the tail tip fasted for eight hours. The FBG was measured by glucose oxidase method. In the principle of safety and effectiveness of dose determination, the safe dose was determined based on the results of previous experiments. The mice in each group were administered intragastrically once a day at the same time for 10 consecutive weeks, based on their body weight.

### 2.4. Determination of GHb, MDA, and SOD in the Blood of Each Group of Mice

The body weight of the mice was measured once a week. FBG values of mice were also measured once a week. After mice were fasted without water for 5 h, blood was collected through the tail vein, and the blood glucose values of each group of mice were measured using the glucose oxidase method. After the last administration, 1 mL of blood was taken from the orbital venous plexus of mice, and a small amount of whole blood was taken immediately for the determination of glycated hemoglobin content by high performance liquid chromatography. The remaining whole blood was centrifuged at 3500 r/min for 15 min, and the supernatant was taken and set aside. Serum SOD and MDA content of each group of mice was determined using ELISA kit.

### 2.5. Collection of Retina Samples

After intraperitoneal injection of 2.5% pentobarbital anesthetized the mice, the blood was taken from the abdominal aorta until the animals went into shock. These mice' eyeballs were removed via ophthalmic scissors and tooth tweezers and placed in 4% paraformaldehyde solution to be fixed for pathological observation and immunohistochemical detection.

### 2.6. Immunohistochemical Staining

The stained specimens were placed under a 400x optical microscope. We randomly selected three high-powered fields of view for each specimen and taken photos using the computer image acquisition system. IPP 6.0 software was used to analyze the optical density of the immunohistochemical photos. The average optical density (integrated optical density/area) was used to represent the relative amount of protein expression, and the mean ± standard deviation was used to analyze the statistical results.

### 2.7. Statistical Methods

All experimental data were processed by SPSS 17.0 statistical software package with the results expressed as mean ± standard deviation. The independent sample *t*-test was used for comparison between the two groups, and one-way analysis of variance was used for comparison of the measurement data among multiple groups. We used one-way ANOVA with post-hoc Tukey HSD test, with the test level of 0.05. *P* < 0.05 indicated that the difference was statistically significant.

## 3. Results

### 3.1. Analysis of the Effective Components of *Coreopsis tinctoria* Nutt

The product of the *Coreopsis tinctoria* Nutt alcohol extract eluted by the macroporous resin was subjected to TLC thin-layer detection and then inspected at 366 nm after unfolding, as shown in Figure 1, and the macroporous resin enriched product was detected by HPLC, as shown in Figure 2. After enrichment with macroporous resin, the content of each component was significantly increased compared with that before purification: chlorogenic acid 26.27 mg/g, flavone mariside 138.50 mg/g, mariside 268.56 mg/g, dicaffeoylquinic acid 16.39 mg/g, brass okaning 83.1 mg/g, and the total content of 532.82 mg/g. Among them, the total flavonoid content of the macroporous resin enrichment products was (in mg/g of naringin) 330 mg/g via ultraviolet detection, significantly higher than that before purification.

#### 3.1.1. Effect of the Effective Components of *Coreopsis tinctoria* Nutt on the Body Weight of db/db Mice

During the whole experiment, the mice in the normal group were in good mental state and moved effortlessly, while the mice in the model group were slow in action and lethargic in spirit. The body weight of the mice was measured every week (Table 1). In terms of body size, the mice in the model group were fatter, and their body weight was significantly higher than that in the normal group, with the difference statistically significant (*P* < 0.05). The body weight of the mice in the drug intervention groups was not significantly different from that in the model group, and the body weight gradually increased with the increase of age.

#### 3.1.2. Effect of the Effective Components of *Coreopsis tinctoria* Nutt on FBG in db/db Mice

By observing the FBG of each group of mice, the experimental results showed (Table 2) that, with the increase in age, the blood glucose level of normal mice gradually increased, but it remained at a normal level. Compared with the normal group of mice, the blood glucose level of the model group was significantly increased, with the difference being statistically significant (*P* < 0.01), and it gradually increased with the increase in age. The blood glucose levels of the mice in the drug intervention groups were lower than those in the model group since week one. The blood glucose level of the positive drug metformin group was also lower than that of the model group mice of the same age, and the difference in week eight was statistically significant (*P* < 0.05). The blood glucose level of the high-dose coreopsis group was lower than that of the model group mice of the same week, and the difference was statistically significant since week four (*P* < 0.05). The blood glucose level of the positive drug plus coreopsis low-dose group had a statistically significant difference since week four (*P* < 0.05).

#### 3.1.3. Effect of the Effective Components of *Coreopsis tinctoria* Nutt on Serum Glycosylated Hemoglobin, MDA, and SOD in db/db Mice

By detecting the glycosylated hemoglobin content in each group of mice, the experimental results showed that (Table 3), compared with the normal group, the serum glycosylated hemoglobin level of the diabetic model group mice was significantly increased (*P* < 0.01). Compared with the model group, the serum glycosylated hemoglobin levels of the drug intervention groups were reduced, where the serum glycosylated levels of the high-dose group and the combination medication group decreased more significantly, and the difference was statistically significant compared with the model group (*P* < 0.01). The observation of the experimental results of the serum MDA level of the mice in each group after the intervention suggested that, compared with the normal group, the serum MDA level of the model group increased significantly (*P* < 0.01). Compared with the model group, serum MDA levels of mice in the metformin group, combination medication group, and high- and low-dose *Coreopsis tinctoria* Nutt groups markedly decreased (*P* < 0.01). Among them, the MDA level of the metformin group decreased most obviously. The observation of the experimental results of the serum SOD content of the mice in each group after the intervention suggested that, compared with the normal group, the serum SOD content of the model group decreased, but the difference was not statistically significant. Compared with the model group, the serum SOD content of mice in the metformin group, combination medication group, and high- and low-dose *Coreopsis tinctoria* Nutt groups increased significantly (*P* < 0.01). Among them, the SOD content of the combination medication group increased most obviously.

#### 3.1.4. Effect of the Effective Components of *Coreopsis tinctoria* Nutt on HE Staining in Retinal Tissue of db/db Mice

As shown in Figure 3, by observing the HE staining slice of retinal tissue under light microscope, the results showed that, in the normal group, the retinal tissue structure had clear hierarchy and orderly arrangement. The ganglion cells were arranged in a single layer with large round or oval nuclei and light staining. The inner layer is thinner, the outer nuclear layer is thicker, the nucleus is smaller, the arrangement is close, and the staining is deeper than the inner layer. In the model group, there were disordered arrangement of ganglion cell layer, sparse arrangement of cells in the inner and outer nuclear layer, vacuole-like changes in cells, and capillary dilatation and congestion. The structure of cells in each layer of retinal tissue was clear and orderly, and the changes of capillary dilatation and congestion were also observed in drug intervention groups.

#### 3.1.5. Effect of the Effective Components of *Coreopsis tinctoria* Nutt on VEGF Expression in the Retina of db/db Mice

As shown in Figure 4, the observation of the VEGF expression in the mice's retinal tissues of each group after the intervention suggested that, compared with the normal group, the VEGF expression in the model group increased significantly (*P* < 0.05). Compared with the model group, the VEGF expressions in each group of drug intervention were reduced. The difference in the single metformin group and the low-dose *Coreopsis tinctoria* Nutt group was statistically insignificant; however, the difference in the low-dose metformin and coreopsis combination group and single high-dose coreopsis was statistically significant (*P* < 0.05), and the decrease in the VEGF expression of in the metformin and coreopsis combination group was the most significant.

#### 3.1.6. Effect of the Effective Components of *Coreopsis tinctoria* Nutt on ICAM1 Expression in the Retina of db/db Mice

As shown in Figure 5, the observation of the ICAM1 expression in the mice's retinal tissues of each group after the intervention suggested that, compared with the normal group, the ICAM1 expression in the model group rose remarkably (*P* < 0.05). Compared with the model group, the ICAM expressions in each drug intervention group decreased. The reduction in the low-dose *Coreopsis tinctoria* Nutt group was the least with the difference statistically insignificant; however, ICAM expressions in the metformin group, low-dose metformin and coreopsis combination group, and high-dose *Coreopsis tinctoria* Nutt group decreased markedly (*P* < 0.05). The reduction in ICAM1 expression in the metformin and coreopsis combination group was the most significant.

#### 3.1.7. Effect of the Effective Components of *Coreopsis tinctoria* Nutt on Bcl-2 Expression in the Retina of db/db Mice

As shown in Figure 6, the observation results of the Bcl-2 expression in the mice's retinal tissues of each group suggested that, compared with the normal group, the Bcl-2 expression in the model group dropped significantly (*P* < 0.05). Compared with the model group, the Bcl-2 expressions in each group of drug intervention increased. The increase in the low-dose *Coreopsis tinctoria* Nutt group was the least obvious, with the difference being statistically insignificant; however, Bcl-2 expressions in the metformin group, low-dose metformin and *Coreopsis tinctoria* Nutt combination group and the high-dose *Coreopsis tinctoria* Nutt group rose significantly (*P* < 0.05), and the increase in ICAM1 expression in the high-dose *Coreopsis tinctoria* Nutt group was the most significant.

#### 3.1.8. Effect of the Effective Components of *Coreopsis tinctoria* Nutt on PEDF Expression in the Retina of db/db Mice

As shown in Figure 7, by observing PEDF expression in the retina of mice in each group, the results showed that, compared with the normal group, the PEDF expression in the model group decreased significantly (*P* < 0.05). Compared with the model group, the PEDF expressions in each group of drug intervention increased. The increase in the low-dose metformin and coreopsis combination group and low-dose *Coreopsis tinctoria* Nutt group was not obvious, with the difference being statistically insignificant; however, the PEDF expressions in the metformin group and the high-dose *Coreopsis tinctoria* Nutt group rose significantly (*P* < 0.05), and the PEDF expression in the high-dose *Coreopsis tinctoria* Nutt group increased most obviously.

## 4. Discussion

Metformin is currently one of the most widely used glucose-lowering drugs in the world, which can reduce blood sugar, regulate blood lipids, improve insulin sensitivity, and prevent the progression of diabetes. Studies have shown that metformin can also improve the fundus lesions of diabetic retinopathy and delay the occurrence and development of diabetes-related vascular complications. A large number of in vitro and in vivo studies and clinical trials have been conducted and are under way. In this study, with stable db/db diabetic mice as the animal model, the experimental results showed that the mice in the normal group were active and agile, while the mice in the model group were slow in action and lethargic in spirit and showed symptoms such as obvious obesity, polydipsia, and polyphagia. Compared with the normal group, the weight of the mice in the model group was significantly higher, while the weight of the mice in the drug intervention groups was not significantly different than that in the model group. Meanwhile, as the week age increases, the weight was on the rise. It is suggested that the effective component extract of *Coreopsis tinctoria* Nutt has no obvious improvement effect on the weight of diabetic mice. The observation of the HE staining of the retinal tissues of each group indicates that the retinal tissue structure in the normal group is clear and ordered. However, in the model group's retinal tissues, there were disordered arrangement of ganglion cell layers, sparse arrangement of in the inner and outer nuclear layer cells, vacuole-like changes in cells, and capillary dilatation and congestion, suggesting that the mice in the model group had suffered early retinopathy damage. In addition, each layer cell of retinal tissue in each drug intervention group is clear in structure and basically orderly in arrangement, with occasionally telangiectasia and congestion, suggesting that the intervention of *Coreopsis tinctoria* Nutt can prevent and delay retinopathy to some extent.

Flavonoids are considered to be the main effective components of the *Coreopsis tinctoria* Nutt. The study by Sha Ailong [10] and others have confirmed that the flavonoids of *Coreopsis tinctoria* Nutt have anti-aging effects, delay atrophy and degeneration of animal organs, promote catabolism, and improve immunity. The study results of Dias et al. [11] have showed that total flavonoids in *Coreopsis tinctoria* Nutt can significantly improve the glucose tolerance of mice, and it is inferred that flavanones and chalcones are the main components from the HPLC/MS component analysis of the effective components. The study results of Xu Bin [12] and others have indicated that kunlun chrysanthemum flavonoid extract has reducing power, free radical scavenging ability, and lipid system antioxidant ability, indicating that kunlun chrysanthemum flavonoid extract boasts more comprehensive antioxidant activity. In the early stage of the research group, the influence of different extracts of *Coreopsis tinctoria* Nutt on the activity of *α*-glucosidase was also discussed, and the results showed that the neutral flavonoids in *Coreopsis tinctoria* Nutt has the strongest inhibitory effect [13]. The total flavonoids in the effective component extract of *Coreopsis tinctoria* Nutt used in this study was 330 mg/g, and its effect on type 2 diabetic mice and retinopathy was observed, which lays a certain theoretical basis for treatment with *Coreopsis tinctoria* Nutt.

In this study, by observing the FBG of each group of mice, the blood glucose level of the model group mice was significantly higher compared with the normal group of mice, with the difference being statistically significant, and it gradually increases according to the disease stage, which become worse with age. The results indicate that the db/db mouse model is stable. Compared with the model group, the serum glycosylated hemoglobin levels of the drug intervention groups were reduced. Among them, the serum glycosylated hemoglobin levels of the high-dose group and the combination medication group decreased more markedly, and the difference is statistically significant compared with the model group. The changes in blood glucose and glycosylated hemoglobin levels are basically the same. The blood glucose and glycosylated hemoglobin levels reflect the overall glucose metabolism state of the body. These results suggest that the high-dose *Coreopsis tinctoria* Nutt group and the combination of Chinese and western drugs have a better control effect on the blood sugar of diabetic mice. In this study, for diabetic mice, the used dosage of metformin, 180 mg/kg BW, merely reduced level of fasting blood glucose at the eighth week. This may be due to the fact that we chose 180 mg/kg as the dose to be administered, which resulted in poor reduction of fasting glucose levels with metformin. In future studies, a dose of 200 mg/kg or even 300 mg/kg, as used by other investigators, could be tried. It also shows that metformin alone has very limited effect in the treatment of diabetes and that it is necessary to combine metformin with other hypoglycemic agents.

The high blood sugar environment in the diabetic state induces the oxidative stress resulting from increase of active oxygen in living cells, which is a common pathogenesis of various diabetic complications. Studies have shown [14] that, with the progression of DR, the serum SOD content shows a trend of gradual decline, suggesting that the occurrence and development of DR is closely related to the reduction of serum SOD content. MDA is a small molecule product produced by lipid peroxidation reaction, which can generate Schiff's base with membrane protein amino acid residues to increase membrane permeability and decrease stability, thereby destroying the structure of cell membranes, causing dysfunction and even death. Therefore, as the currently most representative indicator of body oxidative damage, MDA can reflect the severity of body tissue damage. Studies have shown that MDA plays an important role in the chronic complications of diabetes [15–17].

Through the detection of serum MDA and SOD of mice in each group, the results showed that the SOD level of the combination medication group increased most significantly, and the serum MDA level of mice in the model group increased significantly, with the differences being statistically significant (*P* < 0.01). Among them, the MDA level of the metformin group decreased most significantly. This result suggests that the mice's body in the diabetes model group have experienced oxidative damage, and the *Coreopsis tinctoria* Nutt can significantly improve the oxidative stress state of the body, thus alleviating the oxidative damage to a certain extent. Moreover, the experimental results showed that the effect of the combination medication group was better, suggesting that the combined application of traditional hypoglycemic drugs and traditional Chinese medicine intervention can effectively improve the oxidative damage caused by diabetes, thereby preventing and delaying diabetic complications.

Retinal vascular endothelial growth factor (VEGF) and intercellular adhesion molecule 1 (ICAM1) play an important role in the occurrence and development of DR [18]. After drug intervention, the expressions of VEGF and ICAM1 in the model group increased significantly, while those in the drug intervention groups decreased and that in the metformin and *Coreopsis tinctoria* Nutt combined group decreased most obviously. The results suggest that the effective component extract of *Coreopsis tinctoria* Nutt can prevent and treat diabetic retinopathy by downregulating the expressions of VEGF and ICAM1, and the combination of metformin and *Coreopsis tinctoria* Nutt has a better effect.

Bcl-2 is the first gene to be confirmed to inhibit apoptosis, which is the earliest researched and apoptosis-related proto-oncogene. The occurrence of DR is closely related to apoptosis, whose distinguishing feature is the increase of vascular permeability and pericyte apoptosis [19]. After drug intervention, by observing Bcl-2 expression in the retinal tissues of each group of mice, the Bcl-2 expression in the model group was significantly reduced, while that in each drug intervention group increased, and that in high-dose *Coreopsis tinctoria* Nutt increased most obviously. The results suggest that *Coreopsis tinctoria* Nutt may improve cell apoptosis by upregulating Bcl-2 expression and play a certain role in delaying the occurrence of DR.

Studies have shown that PEDF can inhibit the occurrence and development of DR, which has always been a hot issue of research. During DR, the decreased expression of PEDF may be an important cause of retinal vascular leakage [20]. The current domestic and foreign research can fully illustrate that PEDF has an important protective effect on the retina during DR. By observing PEDF expression in the mice's retina in each group, the PEDF expression in the model group decreased markedly, while that in each drug intervention group increased, with that in the high-dose *Coreopsis tinctoria* Nutt group increased most. This result suggests that *Coreopsis tinctoria* Nutt plays an anti-inflammatory and antioxidant role by upregulating the expression of anti-inflammatory factor PEDF, thus protecting diabetic retina.

In summary, this study used the effective component extract from *Coreopsis tinctoria* Nutt to intervene in the stable db/db diabetic mouse model. It is found that the flavonoids in *Coreopsis tinctoria* Nutt exert the functions as lowering blood sugar and anti-oxidative stress, and the results of the expression of related factors in the retina show that the *Coreopsis tinctoria* Nutt can reduce the expressions of VEGF and ICAM1 and increase the expressions of Bcl-2 and PEDF to give play to its protective effect on DR. The experimental results also show that the combined *Coreopsis tinctoria* Nutt and metformin has a more significant effect on improving the expression of retinopathy-related factors, suggesting that metformin lowered blood sugar while supplementing with *Coreopsis tinctoria* Nutt may be the best way to prevent and treat DR, laying a foundation for the antisugar mechanism and development and utilization of *Coreopsis tinctoria* Nutt in the later period.

## Figures and Tables

**Figure 1:** TLC Atlas of ethanol extract of *Coreopsis tinctoria* Nutt after macroporous resin enrichment (A: marien; B: chlorogenic acid; C: flavanokanin; D: okanin).

**Figure 2:** HPLC Atlas of ethanol extract of *Coreopsis tinctoria* Nutt after macroporous resin enrichment (P2 is chlorogenic acid; P3 and 4 are flavanomarein; P5 is flavanokanin; P9 is marien; P10 is 3,5-dicaffeoyl-quinic acid).

**Figure 3:** HE staining of the tissue of mice retina (GCL: ganglion cell layer; IPL: inner plexiform layer; INL: inner nuclear layer; OPL: outer plexiform layer; ONL: outer nuclear layer; DA: disordered arrangement; SA: sparse arrangement; DAC: dilatation and congestion).

**Figure 4:** Immunohistochemistry observation of VEGF expression in retina of mice (^∗^*P* < 0.05 versus normal group; ^#^*P* < 0.05 versus model group).

**Figure 5:** Immunohistochemistry observation of ICAM1 expression in retina of mice (^∗^*P* < 0.05 versus normal group; ^#^*P* < 0.05 versus model group).

**Figure 6:** Immunohistochemistry observation of Bcl-2 expression in retina of mice (^∗^*P* < 0.05 versus normal group; ^#^*P* < 0.05 versus model group).

**Figure 7:** Immunohistochemistry observation of PEDF expression in retina of mice (^∗^*P* < 0.05 versus normal group; ^#^*P* < 0.05 versus model group).

**Table 1:** Changes of body weight of db mice (g).

	NG	DC	DC + M	DC + M + EC	DC + EC150	DC + EC300
Initial level	16.8 ± 0.46	30.4 ± 1.63^*∗∗*^	30.61 ± 0.83	30.61 ± 0.69	30.81 ± 1.74	30.64 ± 1.42
Week 1	19.5 ± 0.36	33.4 ± 2.11^*∗∗*^	32.44 ± 0.9	33.15 ± 0.75	33.35 ± 1.79	32.93 ± 1.47
Week 2	20.89 ± 0.4	34.0 ± 2.41^*∗∗*^	33.02 ± 1.06	33.84 ± 1.05	34.51 ± 2.05	33.53 ± 1.6
Week 3	21.5 ± 0.40	34.7 ± 2.46^*∗∗*^	33.27 ± 1.25	34.83 ± 1.35	35.58 ± 2.28	34.04 ± 1.65
Week 4	21.2 ± 0.31	34.3 ± 2.61^*∗∗*^	34.03 ± 1.51	35.17 ± 1.64	37.31 ± 2.54	34.68 ± 2.00
Week 5	23.3 ± 0.45	36.7 ± 2.79^*∗∗*^	36.28 ± 1.64	37.61 ± 1.70	39.14 ± 2.78	35.86 ± 2.33
Week 6	23.4 ± 0.45	36.7 ± 2.95^*∗∗*^	37.32 ± 1.74	38.58 ± 1.95	39.44 ± 2.96	36.65 ± 2.46
Week 7	23.8 ± 0.51	37.6 ± 3.02^*∗∗*^	38.11 ± 1.73	39.44 ± 2.07	39.48 ± 3.08	38.00 ± 2.65
Week 8	23.8 ± 0.50	37.0 ± 3.29^*∗∗*^	38.69 ± 1.81	38.98 ± 2.10	39.76 ± 3.09	38.25 ± 2.83
Week 9	24.3 ± 0.46	38.3 ± 3.59^*∗∗*^	39.73 ± 1.95	39.81 ± 1.94	41.08 ± 3.40	40.59 ± 3.05

Values were expressed as mean ± SD; ^∗∗^*P* < 0.01 versus normal group.

**Table 2:** Changes of FBG of db mice (mmol/L).

	NG	DC	DC + M	DC + M + EC	DC + EC150	DC + EC300
Week 1	4.26 ± 0.22	9.34 ± 0.98^*∗∗*^	8.39 ± 0.33	8.00 ± 1.04	7.45 ± 0.56	8.18 ± 0.78
Week 2	4.14 ± 0.13	11.2 ± 0.88^*∗∗*^	10.91 ± 0.99	9.97 ± 0.83	10.83 ± 1.01	10.04 ± 1.04
Week 3	6.81 ± 0.27	14.1 ± 1.44^*∗∗*^	11.83 ± 1.46	11.47 ± 1.18	11.49 ± 1.61	11.02 ± 1.54
Week 4	5.24 ± 0.42	14.0 ± 1.94^*∗∗*^	13.83 ± 1.48	9.79 ± 1.82^#^	13.24 ± 1.81	9.92 ± 1.15^#^
Week 5	4.67 ± 0.30	12.7 ± 1.44^*∗∗*^	10.85 ± 1.18	9.60 ± 1.30^#^	10.44 ± 1.33	9.62 ± 0.81^#^
Week 6	5.17 ± 0.21	12.1 ± 1.47^*∗∗*^	9.48 ± 1.40	9.05 ± 1.26^#^	9.88 ± 1.30	9.29 ± 0.84^#^
Week 7	5.59 ± 0.38	16.5 ± 2.26^*∗∗*^	13.13 ± 1.24	11.97 ± 1.77^#^	13.91 ± 1.28	12.6 ± 1.81^#^
Week 8	7.68 ± 0.42	17.1 ± 1.96^*∗∗*^	12.82 ± 1.64^#^	12.41 ± 1.15^#^	14.93 ± 1.31	11.1 ± 1.31^##^
Week 9	7.95 ± 0.50	19.0 ± 2.00^*∗∗*^	14.58 ± 2.00	13.62 ± 1.90^#^	16.75 ± 1.80	13.6 ± 1.60^#^

Values were expressed as mean ± SD; ^∗∗^*P* < 0.01 versus normal group; ^#^*P* < 0.05, ^##^*P* < 0.01 versus model group.

**Table 3:** The level of serum GHb (%), MDA (mmol/mL), and SOD (U/mL) in db mice.

	NG	DC	DC + M	DC + M + EC	DC + EC150	DC + EC300
GHb	4% ± 0.0	7.6% ± 1.0^*∗∗*^	7.2% ± 1.3	6.4% ± 0.9^##^	6.9% ± 1.3	6.4 ± 1.1^##^
MDA	6.857 ± 1.253	10.28 ± 1.938^*∗∗*^	5.016 ± 0.679^##^	5.200 ± 0.580^##^	6.476 ± 0.917^##^	5.086 ± 0.778^##^
SOD	188.42 ± 32.99	159.04 ± 36.05	326.68 ± 76.47^#^	440.59 ± 55.89^#^	295.88 ± 93.16^#^	416.95 ± 68.46^#^

Values were expressed as mean ± SD; ^∗^*P* < 0.05, ^∗∗^*P* < 0.01 versus normal group; ^#^*P* < 0.05, ^##^*P* < 0.01 versus model group.

## Data Availability

The datasets used and/or analyzed during the current study are available from the corresponding author on reasonable request.
